# Effectiveness of Nursing Risk Management in Neonatal Asphyxia Resuscitation Care

**DOI:** 10.1155/2022/5465472

**Published:** 2022-06-03

**Authors:** Zhen Ye, Wenjun Wang, Peili Sun

**Affiliations:** ^1^Delivery Room, People's Hospital of Lujiang County, Lujiang County, Hefei 231500, Anhui Province, China; ^2^People's Hospital of Lujiang County, Lujiang County, Hefei 231500, Anhui Province, China; ^3^Department of Infectious Diseases, People's Hospital of Lujiang County, Lujiang County, Hefei 231500, Anhui Province, China

## Abstract

**Objective:**

To analyze the effectiveness of nursing risk management in neonatal asphyxia resuscitation care and to observe and summarize the nursing measures and outcomes.

**Methods:**

A total of 60 neonatal asphyxia cases from January 2021 to December 2021 were recruited and assigned via a random number table method at a ratio of 1 : 1 to receive either routine care plus nursing risk management (the observation group, *n* = 30) or routine care (the control group, *n* = 30). Outcome measures included blood gas index, neonatal Apgar score, neonatal behavioral neurological assessment (NBNA) score, nursing satisfaction, and complications.

**Results:**

The differences in partial pressure of oxygen (PaO_2_) and partial pressure of carbon dioxide (PaCO_2_) between the two groups before care were not statistically significant (*P* > 0.05), while after care, PaO_2_ in the observation group had a higher level of PaO_2_ and a lower level of PaCO_2_ than the control group (*P* < 0.01). The two groups showed similar Apgar scores and NBNA scores before care (*P* > 0.05), while after care, routine care plus nursing risk management resulted in higher Apgar scores and NBNA scores versus routine care alone (*P* < 0.01). The nursing satisfaction rate in the observation group (96.67%) was significantly higher than that of the control group (73.33%) (*P*=0.030). Nursing risk management plus routine care was associated with a significantly lower incidence of complications (6.67%) compared to routine care (26.67%) (*P*=0.038).

**Conclusion:**

Nursing risk management in neonatal asphyxia resuscitation care showed outstanding outcomes in improving neonatal blood gas index, neurological function, and Apgar score, while reducing the occurrence of complications and achieving high nursing satisfaction.

## 1. Introduction

As common neonatal complication [1], neonatal asphyxia refers to the difficulty of the fetus in breathing normally or regularly within 1 min after delivery [2], with specific presentations including weakened breath, blue skin, slowed heart rate, limb flaccidity, and scarce reflexes. It is a major contributor to neonatal death and mental retardation [3]. Epidemiological studies have found that 1/4 of the neonatal deaths worldwide each year are attributed to neonatal asphyxia [4], and its incidence is on the rise with the increase in advanced maternal age and changes in the environment [5]. Nursing risk is the possibility of patient injury or death due to uncertainties in the nursing process [3], and nursing risk management is a management approach to identify and assess these uncertainties to avoid risk events and realize maximum safety [5]. The anticipatory factors of neonatal asphyxia are complex, and ineffective treatment is associated with severe adverse outcomes. Active resuscitation care for neonatal asphyxia in clinical practice is of great importance to improve survival rates [6]. Traditional care of neonatal asphyxia mainly focuses on monitoring, respiratory management, and resuscitation cooperation, and it lacks pertinency and risk awareness. Nursing risk management has been applied in neonatal asphyxia resuscitation care and allows the development of preventive and intervention measures to reduce complications [7]. The clinical manifestations of neonatal asphyxial brain damage are similar to those of “Pixue Neibi” (blood stagnation) in traditional Chinese medicine, and its pathogenesis is stagnation of blood in the brain and obstruction of blood vessels and channels. Danshen injection is effective in relieving asphyxiated cerebral edema, preventing secondary intracranial pressure increase, reducing existing brain damage, and preventing new brain damage. To investigate the value of nursing risk management, this study recruited 60 cases of neonatal asphyxia in our hospital for analysis.

## 2. Materials and Methods

### 2.1. General Information

Sixty cases of neonatal asphyxia from January 2021 to December 2021 were recruited and assigned via a random number table method at a ratio of 1 : 1 to receive either routine care plus nursing risk management (the observation group, *n* = 30) or routine care (the control group, *n* = 30). In the observation group, there are 16 male infants and 14 female infants with an average gestation period of 38.59 ± 2.32 weeks (35–40 weeks), birth weight of 2324 g–3842 g, and mean weight of 2894.28 ± 323.68 g. There were 21 cases of mild asphyxia and 9 cases of severe asphyxia in terms of disease severity and 22 cases of vaginal delivery and 8 cases of cesarean delivery in terms of the delivery mode. In the control group, there were 17 male infants and 13 female infants with an average gestation period of 38.31 ± 2.37 weeks (36–41 weeks), birth weight of 2405 g–3850 g, and mean weight of 2915.52 ± 305.72 g. There were 21 cases of mild asphyxia and 9 cases of severe asphyxia in terms of disease severity and 22 cases of vaginal delivery and 10 cases of cesarean delivery in terms of the delivery mode. The baseline characteristics of the two groups were comparable (*P* > 0.05). The families of the included infants provided written informed consent after being informed of the study purpose and study procedure. This study was approved by the medical ethics committee of People's Hospital of Lujiang County, no. 59873.

### 2.2. Inclusion and Exclusion Criteria

Inclusion criteria were as follows: (1) infants who were diagnosed as neonatal asphyxia by X-ray, head ultrasound, and CT [8] with an Apgar score of <7 points at 1 min after birth; who received cardiopulmonary resuscitation treatment; with complete data and no major organic diseases; with complete clinical examination data were included. Exclusion criteria were as follows: (1) infants with seriously damaged important organs; with congenital heart disease; with systemic infectious diseases; with other types of neonatal complications; with abnormal immune function or coagulation disorders; with respiratory system or central nervous system pathologies; and with hemorrhagic shock were excluded. Elimination criteria were as follows: (1) those with missing clinical data; with severe life-threatening complications during the study; and with the withdrawal of consent were excluded.

### 2.3. Methods

In the control group, conventional nursing interventions were performed, and resuscitation was given to newborns. The ABCD process was followed to construct respiratory channels and maintain the neonate's airway open. Chest compressions and drug treatment following medical prescription were also applied, and the newborn was kept warm during the whole treatment process. The temperature of the thermal radiation table was adjusted to 32°C–34°C. A similar conventional nursing protocol was introduced to patients in the observation group.

The subjects in the observation group additionally received nursing risk management. (1) A nursing risk management team for neonatal asphyxia composed of experienced head nurses, specialist nurses, and key nurses was established, and the risk factors related to the care of neonatal asphyxia were comprehensively analyzed. The nurses' cognition and management skills of neonatal asphyxia were strengthened, and resuscitation drills were conducted to improve emergency response and nursing capabilities. (2) Preresuscitation assessment: maternal, physical, and mental conditions were comprehensively monitored to keep track of maternal comorbidities, the progress of labor, and other relevant factors, with an assessment of the risk of neonatal asphyxia and preparation of resuscitators, masks, oxygen, and other emergency equipment in advance. Medical and nursing staffs were aware of their respective duties and performed accordingly to ensure smooth resuscitation. (3) Nursing during resuscitation: a 3 cm–5 cm umbilical cord should be appropriately retained during severing, to allow for subsequent umbilical vein cannulation and shorten the peripheral venous time, so as to gain time for neonatal resuscitation and increase the success rate. The newborn was kept warm on a preheated warming table, the blood and amniotic fluid on the body surface of the infant were removed, and the umbilical temperature was maintained at about 36°C-37°C. (4) Neonatal monitoring: the newborn's body temperature, pulse, and skin color were closely monitored, and any abnormalities were reported promptly to the physician for corresponding treatment. (5) Airway management: the newborn was put in a lateral position, with the head and chest appropriately padded at 15°–20°, to avoid vomit from entering the airway and to maintain respiratory flow. The respiratory tract was cleared, and back-patting and sputum suction were performed if necessary. In the event of no response from the newborn, tracheal intubation was performed for resuscitation. (6) Disinfection management: in strict accordance with aseptic operation, the ward and resuscitation room were thoroughly disinfected with good ventilation and control of the number of visitors to prevent cross-infection.

The subjects received 0.4 ml per kg (body weight) of Danshen injection (diluted in 10 mL of 10% glucose injection) and 30 mg per kg (body weight) of vitamin C (diluted in 10 mL of 10% glucose injection) through an intravenous drip, with a dripping rate of 4-5 drops per minutes, twice daily. The duration of treatment was 10 days.

### 2.4. Observation Indexes

The improvement of neonatal blood gas indexes before and after care were monitored, the changes in neonatal health status and neurological function before and after care were assessed, nursing satisfaction was obtained with a self-prepared questionnaire, and the occurrence of any complications were followed-up and recorded. (1) Blood gas indexes, including partial pressure of oxygen (PaO_2_) and partial pressure of carbon dioxide (PaCO_2_), were determined with a Wofen GEM3500 automatic blood gas analyzer (Nanjing Hanyuyiliao Technology Co., Ltd.). (2) An Apgar score was used to assess the health status of newborns, mainly involving heart rate, breathing, muscle tone, laryngeal reflex, and skin color, with a total score of 10 points. A score of <7 points indicates the presence of asphyxia and of <4 points indicates severe asphyxia. The higher the score, the better the health status [9]. (3) The neonatal behavioral neurological assessment (NBNA) score was used to assess neonatal neurological function, which consisted of 20 items in 5 dimensions, and each item scored 0–2 points. The score range was 0–40 points, and a higher score indicated better neurological function [10]. (4) The nursing satisfaction questionnaire, self-developed by our department, included 20 question items, and each item was scored 0–5 points, with a total score of 100 points. A score of ≥80 points indicates highly satisfied, 60–79 points indicates satisfied, and <60 points indicates dissatisfied. (5) Complications included intracranial hemorrhage, apnea, hypoxic encephalopathy.

### 2.5. Statistical Methods

Data analyses were performed on the SPSS22.0 software package. The counting data are expressed as (%) and analyzed using the chi-square test, and the measurement data are expressed as (mean ± SD) and analyzed using the Student's *t*-test. The test results were evaluated with 0.05 as the threshold, and a *P* value less than 0.05 indicated that the difference between groups was statistically significant.

## 3. Results

### 3.1. Comparison of Blood Gas Indexes between the Two Groups of Neonates

After nursing, PaO_2_ levels increased, and PaCO_2_ levels decreased significantly (*P* < 0.01). The intergroup comparison showed that the observation group had lower PaCO_2_ levels and higher PaO_2_ levels than the control group (*P* < 0.01) (Table 1).

### 3.2. Comparison of Apgar Scores and NBNA Scores of Neonates in the Two Groups

The two groups showed similar Apgar scores and NBNA scores before care (*P* > 0.05), while after care, routine care plus nursing risk management resulted in higher Apgar scores and NBNA scores versus routine care alone (*P* < 0.01) (Table 2).

### 3.3. Comparison of Satisfaction between the Two Groups

The nursing satisfaction rate in the observation group (96.67%) was significantly higher than that of the control group (73.33%) (*P*=0.030) (Table 3).

### 3.4. Comparison of Complications between the Two Groups

Nursing risk management plus routine care was associated with a significantly lower incidence of complications (6.67%) compared to routine care (26.67%) (*P*=0.038) (Table 4).

## 4. Discussion

Neonatal asphyxia is a state of hypoxia in which the fetus is delivered with abnormal respiratory and circulatory disorders and fails to breathe on its own. It features a high incidence and is one of the major causes of neonatal death, cerebral palsy, and mental retardation [11]. Research has found that hypoxia is the main factor leading to neonatal asphyxia, and rapid and accurate resuscitation is required to keep the newborn's airway open for the onset of neonatal asphyxia [12]. Neonatal asphyxia is associated with gas exchange disorders and a cascade of complications, such as hypercapnia, hypoxemia, and hypoxic-ischemic encephalopathy [13]. Numerous clinical studies have confirmed that nursing risk management in the resuscitation care of neonatal asphyxia contributes to safeguarding children's health and reducing disability and mortality. However, nursing risk management places higher demands on nursing staff which indicates more training and medical costs. The level of neonatal asphyxia resuscitation techniques has been improving as recent health care technology advances, which is of great significance in reducing neonatal mortality and improving the quality of life of patients.

In addition to necessary clinical treatment and resuscitation, nursing interventions are essential to reduce mortality and enhance the prognosis of neonatal asphyxia. Conventional care of neonatal asphyxia mainly focuses on disease observation and resuscitation, which lacks foresight and has a poor emergency response. As a new nursing management model, nursing risk management accurately and effectively identifies potential risk factors and uncertainties in nursing work and formulates relevant countermeasures in advance, which reduces the damage to the children and ensures nursing safety. Nursing risk management transforms passive care into active care. The results of the present study showed that risk nursing management was associated with significantly better blood gas indices versus routine care, indicating that nursing risk management improved the blood gas of the children. Infection is the most common complication of neonatal asphyxia, which is attributed to improper aseptic operation and inadequate disinfection. Therefore, disinfection management should be strengthened for infection prevention to avoid cross-infection, pulmonary infection, and other related complications. As neonatal asphyxia is often accompanied by hypothermia, nursing staff should enhance their understanding of its risk factors and strengthen thermal care. Early risk management and proper care reduce the incidence of ischemic-hypoxic encephalopathy and improve the neurological function of children. In the present study, risk nursing management resulted in significantly higher Apgar scores in patients and a lower incidence of complications versus routine care, suggesting that the application of nursing risk management improves neonatal health status and reduces the damage to neurological function. Nursing risk management is patient-centered and proactively assesses potential risk factors based on the actual clinical situation of the patient to formulate corresponding contingency plans and specific treatment measures to restrain all potential risks, which greatly improves the quality of care. Previous studies have reported that risk management could reduce nurse-patient disputes, enhance the prognosis of the child, and promote nursing satisfaction. In the present study, the nursing satisfaction of the observation group was higher than that of the control group, indicating that the families of these infants were satisfied with this nursing method.

Treatment with Danshen injection and vitamin C for neonatal asphyxia improves the recovery, reduces sequelae, shortens the duration of treatment, and decreases the frequency and dosage of continuous antispasmodics. Vitamin C can remove excessive free radicals produced during hypoxic brain damage, and Danshen injection can improve microcirculation, enhance brain tissue metabolism and regulation, and repair damaged brain cells, thereby improving the therapeutic effect and reducing sequelae. The current issues in risk nursing management include the enhancement of the training of asphyxia resuscitation personnel and further perfection of evaluation indicators of successful resuscitation of asphyxiated newborns.

## 5. Conclusion

Nursing risk management in neonatal asphyxia resuscitation care showed outstanding outcomes in improving neonatal blood gas index, neurological function, and Apgar score, while reducing the occurrence of complications and achieving high nursing satisfaction. The limitation of this study is the absence of long-term follow-up of children and regular monitoring of their intelligence to support the effectiveness of this care strategy. Future studies with long-term follow-up are required to provide more reliable data for clinical references.

## Figures and Tables

**Table 1:** Comparison of blood gas indexes between the two groups of neonates (mmHg, $\bar{x}$ ± *s*).

Group	Number of cases	PaO_2_		PaCO_2_	
		Precare	Aftercare	Precare	Aftercare
Observation group	30	47.14 ± 4.73	78.12 ± 6.94^*∗*^	54.26 ± 5.64	41.75 ± 3.15^*∗*^
Control group	30	46.24 ± 5.59	65.16 ± 5.46^*∗*^	55.37 ± 6.58	48.14 ± 4.36^*∗*^
*t*	—	0.673	8.039	0.702	6.507
*P*	—	0.504	**<0.01**	0.486	**<0.01**

Note: compared with precare,^*∗*^*P* < 0.05.

**Table 2:** Comparison of Apgar scores and NBNA scores of neonates in the two groups (scores, $\bar{x}$ ± *s*).

Group	Number of cases	Apgar score		NBNA score	
		Precare	Aftercare	Precare	Aftercare
Observation group	30	6.22 ± 1.20	9.83 ± 0.25^*∗*^	27.48 ± 2.43	38.42 ± 3.32^*∗*^
Control group	30	6.35 ± 1.15	8.42 ± 0.16^*∗*^	26.93 ± 2.12	33.53 ± 3.25^*∗*^
*t*	—	0.428	26.019	0.934	5.765
*P*	—	0.670	**<0.01**	0.354	**<0.01**

Note: compared with precare, ^*∗*^*P* < 0.05.

**Table 3:** Comparison of satisfaction between the two groups (%).

Group	Number of cases	Very satisfied	Basically satisfied	Dissatisfied	Nursing satisfaction (%)
Observation group	30	23 (76.67)	6 (20.00)	1 (3.33)	29 (96.67)
Control group	30	16 (56.67)	6 (20.00)	8 (26.67)	22 (73.33)
*X* ^2^	—	—	—	—	4.706
*P*	—	—	—	—	0.030

**Table 4:** Comparison of complications between the two groups (%).

Group	*n*	Intracranial hemorrhage	Apnea	Anoxic encephalopathy	Incidence of complications (%)
Observation group	30	1 (3.33)	0 (0.00)	1 (3.33)	2 (6.67)
Control group	30	2 (6.67)	3 (10.00)	3 (10.00)	8 (26.67)
*X* ^2^	—	—	—	—	4.320
*P*	—	—	—	—	0.038

## Data Availability

All data generated or analysed during this study are included in this published article.
